The article "Intelligent Image Diagnosis of Pneumoconiosis Based on Wavelet Transform-Derived Texture Features" was published in 2022. Journal: Comput Math Methods Med.

# Intelligent Image Diagnosis of Pneumoconiosis Based on Wavelet Transform-Derived Texture Features

**DOI:** 10.1155/2022/2037019

**Published:** 2022-03-17

**Authors:** Zichen Wang, Maoneng Hu, Min Zeng, Guoliang Wang

**Affiliations:** Department of Imaging, The Third Clinical College of Hefei of Anhui Medical University, The Third People's Hospital of Hefei, Hefei 230022, China

## Abstract

**Objective:**

Early diagnosis and treatment of occupational pneumoconiosis can delay the development of the disease. This study is aimed at investigating the intelligent diagnosis of occupational pneumoconiosis by wavelet transform-derived entropy.

**Method:**

From June 2013 to June 2020, the high KV digital radiographs (DR) and computed tomography (CT) images from a total of 60 patients with occupational pneumoconiosis in our department were selected. The wavelet transform-derived texture features were extracted from all images, and the decision tree was used for feature selection. The support vector machines (SVM) with three kernel functions were selected to classify the two kinds of images, and their diagnostic efficiency was compared.

**Result:**

After eight times of wavelet decomposition, eight wavelet entropy texture features (feature set) were extracted, and six were selected to form the feature subset. The classification effect of linear kernel function SVM is better than those of other functions, with an accuracy of 84.2%. The diagnostic values of DR and CT for occupational pneumoconiosis were the same (kappa = 0.737, *P* < 0.001). The detection rate of CT for stage I of occupational pneumoconiosis was significantly higher than that of DR (*P* = 0.031).

**Conclusion:**

It is helpful to improve the early diagnosis level of pneumoconiosis by using SVM to make an intelligent diagnosis based on the wavelet entropy.

## 1. Introduction

Occupational pneumoconiosis is a systemic disease caused by diffuse fibrosis in lung tissue caused by long-term inhalation of productive dust and occupation during occupation activities [1–3]. Its pathogenesis is complex, and the primary process is as follows: when dust particles enter the upper respiratory tract and alveoli, about 2%~3% of them will eventually deposit in the alveolar wall; then, it will be phagocytized and digested by macrophages in human tissues; finally, the particles discharged from the body or transported to the lymphatic system [4]. When the human body inhales a large number of free silica particles, the latter accumulates in the alveolar wall [5]. Pneumoconiosis has the characteristics of occult and long incubation period, which can not be cured and can be aggravated year by year [6]. Although the incidence of pneumoconiosis is decreasing overall, the incidence rate of some special causes, such as asbestosis, is rising [7]. After a long period of inflammatory stimulation, pneumoconiosis is highly likely to develop into mesothelioma [8].

The article "Intelligent Image Diagnosis of Pneumoconiosis Based on Wavelet Transform-Derived Texture Features" was published in 2022. Journal: Comput Math Methods Med.

Early diagnosis and treatment of occupational pneumoconiosis can delay the development of the disease. At present, the diagnosis and staging of occupational pneumoconiosis in China are mainly based on the high KV X-ray and the posteroanterior digital radiography (DR) [9]. Computed tomography (CT) and magnetic resonance imaging (MRI) were also used to diagnose pneumoconiosis. However, due to the scanning time and resolution, MRI is difficult to be used as a routine examination method [10, 11]. Due to the complexity and diversity of X-ray manifestations of pneumoconiosis, it is challenging to master the classification criteria. The accuracy of early diagnosis of pneumoconiosis needs to be improved. The results show small shadows with different sizes, uneven distribution, and densities in pneumoconiosis patients' images, which show different texture characteristics from healthy people's DR chest films. In medical images, the quantitative or qualitative changes of texture features often reflect the pathological changes of the body. Therefore, researchers try to use a variety of texture analysis techniques to analyze various medical imaging images and explore new ways of disease diagnosis and treatment. Due to the complexity of medical images and their textures, there is no general texture analysis method suitable for all kinds of medical images.

In recent years, wavelet transform has been widely used in image processing [12–15]. Because wavelet transform can concentrate the energy of the original image on a small number of wavelet coefficients and the decomposed wavelet coefficients have a high local correlation in the detail components of three directions, it provides favorable conditions for feature extraction. At present, some researchers have applied the features of energy and entropy based on wavelet transform to the texture analysis of ceramic tiles and textiles and achieved good results [16, 17]. As the city's occupational disease prevention and control hospital, our hospital has carried out the research and development of the accurate diagnosis of occupational pneumoconiosis with multimodal imaging. In this study, the value of wavelet entropy texture features for pneumoconiosis diagnosis was applied. The aim is to improve the early diagnosis and differential diagnosis of occupational pneumoconiosis.

## 2. Materials and Methods

### 2.1. Research Objects

A total of 120 imaging data were from the Department of Radiology, the Third People's Hospital of Hefei. All patients were male. Specifically, 60 were healthy persons received physical examination, and the rest were 60 patients with pneumoconiosis. All patients were male, aged 33-86 years, with an average of 52.18 ± 14.11 years. They had a dust exposure history of 4-30 years, with an average of 11.85 ± 6.76 years. The main symptoms were chronic cough, expectoration, chest pain, chest tightness, shortness of breath, dyspnea, etc.

The article "Intelligent Image Diagnosis of Pneumoconiosis Based on Wavelet Transform-Derived Texture Features" was published in 2022. Journal: Comput Math Methods Med.

### 2.2. Inspection Method

Digital X-ray imaging system (DXR vision) produced by Neusoft company was used for chest high KV DR examination. Take the standard chest posteroanterior position; imaging parameters were set as 120~140 kV, power≧20 kW, 4~8 mAs, exposure time≦0.1 s, focus≦1.2 mm, and focal film distance of 1.8 m. The patient's chest wall was close to the detector, the feet were naturally separated, and the arms rotate inward so that the scapula does not overlap with the lung field. The centerline was aligned with the height of the sixth thoracic vertebrae, and the exposure is conducted under a breath holding state after full deep inspiration.

The chest CT scan was performed with optima CT produced by GE company. The imaging parameters were 120 kV and 200 mAs. The patient was supine on the examination table with both arms raised. The patient was positioned at the level of sternal stalk notch. The chest was positioned in a positive position. The scanning range was 2-3 cm from the apex of the lung to the diaphragm. Thin layer scanning was used for the local lung field with suspected abnormalities or small lesions. The interval between layers was 1.25 mm, and the thickness was 1.25 mm. The bone algorithm was used for reconstruction.

Furthermore, the original image was saved in terms of DICOM. Then, the lung fields was extracted from the imaging data after image enhancement via the most significant between-class variance algorithm based on morphological reconstruction.

### 2.3. Wavelet Texture Features

The texture of the pneumoconiosis imaging data was different from those of the normal ones because there were a certain number of small shadows in the pneumoconiosis imaging data, which could not be found in the normal ones. Based on this, a diagnosis of pneumoconiosis could be made. This paper, therefore, performed wavelet decomposition based on db7 wavelet basis and calculated the entropy of wavelet coefficients as texture features. Furthermore, the definition and calculation process of wavelet entropy is as follows.

Assuming that N-level wavelet decomposition was performed, the *K*-th wavelet coefficient sequence of the *i* (*i* = *l*, 2, ⋯, *N*) decomposition layer was recorded as {*S*_*ik*_ | (*k* = 1,2,3, ⋯)}. Meanwhile, let *E*_*i*_ be the energy of the *i* decomposition layer on the *k* scale; then,

(1) $$\begin{array}{c} E_{i}=\underset{k=1}{\sum }S_{ik}^{2}. \end{array}$$

Use the total energy *E* of the image (that is, the sum of the energy *E*_*i*_ of each layer) to normalize the energy *E* of the *i* decomposition layer to obtain the relative energy *P*_*i*_ of the *i* decomposition layer, that is,

(2) $$\begin{array}{c} p_{i}=\frac{E_{i}}{E}. \end{array}$$

According to Shannon's information entropy theory, the wavelet entropy *H*_*i*_ of the *i* decomposition layer was defined as

(3) $$\begin{array}{c} H_{i}=-p_{i}\ln p_{i}. \end{array}$$

According to the size of the DR image, 8 wavelet decompositions were performed on the image, finally obtaining a feature vector composed of 8 wavelet entropy values:

(4) $$\begin{array}{c} H=\left[H_{1},H_{2},H_{3},H_{4},H_{5},H_{6},H_{7},H_{8}\right]. \end{array}$$

The article "Intelligent Image Diagnosis of Pneumoconiosis Based on Wavelet Transform-Derived Texture Features" was published in 2022. Journal: Comput Math Methods Med.

### 2.4. Feature Selection Based on Decision Tree

Since the wavelet transform was performed layer by layer on the same image, there would be a certain correlation between the texture features based on the wavelet transform, thus generating redundant features. In addition, there might be noise features interfering with the classification process of the classifier. Therefore, before using wavelet entropy for pneumoconiosis diagnosis and classification, the decision tree was first employed for feature selection.

The decision tree algorithm finds the feature with the best classification ability and divides the data into multiple subsets. Each subset was divided by the feature with the best classification ability until the condition for the decision tree to stop growing was met. Therefore, the result of decision tree feature selection was those features considered to have the best classification ability in each subset. According to the criteria for judging the ability of feature classification, there were many growth algorithms for decision trees, such as the ID3 algorithm based on information entropy, the CART algorithm based on Gini index, the C4.5 algorithm based on information gain rate, and the C5.0 algorithm. Considering that wavelet entropy was all continuous features, this paper applied C5.0 algorithm decision tree to feature selection.

### 2.5. Support Vector Machine Classifier

From the perspective of data mining, disease diagnosis was a binary classification task; therefore, an appropriate classifier model should be selected for pneumoconiosis diagnosis via texture features of imaging data. The support vector machine (SVM) was a research direction in statistical learning. It was developed based on the theory of small sample statistics and possessed a positive generalization ability for high-dimensional spaces. What is more, for the second-class data classification problem, the basic idea of SVM was to find an optimal hyperplane via a kernel function to maximize the gap between the two categories. Furthermore, the performance of SVM is closely related to the choice of the kernel function. Accordingly, an SVM classifier with good generalization ability could obtain only by selecting a suitable kernel function and projecting the data into a suitable feature space.

The article "Intelligent Image Diagnosis of Pneumoconiosis Based on Wavelet Transform-Derived Texture Features" was published in 2022. Journal: Comput Math Methods Med.

There are many kernel functions of support vector machines, and there is no established standard to judge the applicability of kernel functions. Therefore, this study selected the following three kernel functions for comparative research.

1. Linear kernel function:

(5) $$\begin{array}{c} K\left(x,y\right)=x∙y. \end{array}$$

(2) Polynomial kernel function:

(6) $$\begin{array}{c} K\left(x,y\right)={\left(x∙y+1\right)}^{q},q=1,2,\cdots ,N. \end{array}$$

(3) Gaussian kernel function:

(7) $$\begin{array}{c} K\left(x,y\right)=\exp\left\{-\frac{{\left|x-y\right|}^{2}}{2\sigma^{2}}\right\}. \end{array}$$

Among them, *x* is the input feature vector, the category of which is *y* ∈ {0, 1}, and *q* is the degree of the polynomial. Moreover, in this paper, *q* = 3; the learning parameter *σ*^2^ is used to determine the distance between sample vectors in the feature space in accordance with the empirical text, *σ*^2^ = 0.1. Additionally, the output of the SVM is a decimal *C* between 0 and 1, and it is divided into two categories with a limit of 0.5. That is, a sample with *C* ≥ 0.5 is diagnosed as a pneumoconiosis patient, while a diagnosis with *C* < 0.5 is a normal person.

### 2.6. Evaluation of the Classifier Model

When verifying the SVM model, considering the number of sample cases and the time of calculation, a 5-fold cross validation method was employed. Specifically, all imaging data were randomly divided into 5 subsets, each of which included 7 normal imaging data and 5 imaging data of pneumoconiosis patients. Furthermore, in a certain round of model verification, 4 sample subsets were used as the training set to train the model, and the remaining 1 sample subset was used as the test set to verify the model. Then, after 5 rounds of modeling-testing, the SVM output for classifying all imaging data was saved, and the classification accuracy, sensitivity, and specificity were calculated. What is more, the receiver operating characteristic (ROC) and the area under the curve (AUC) represented the average specificity of the classification results under various specificities or displayed the average sensitivity of the result under various sensitivities. Accordingly, it was used as a comprehensive index to evaluate the SVM classification results.

The article "Intelligent Image Diagnosis of Pneumoconiosis Based on Wavelet Transform-Derived Texture Features" was published in 2022. Journal: Comput Math Methods Med.

### 2.7. Observation Index

The total detection rate and the detection rate for variant stages of occupational pneumoconiosis were compared by high KV DR and CT and the detection of pulmonary complications.

### 2.8. Statistical Analysis

The normality of data was tested by the Kolmogorov-Smirnov method and Shapiro-Wilk method. If the *P* values were larger than or equal to 0.05, the data conform to normal distribution. The measurement data was expressed by $\bar{x}\pm s$, and the statistical analysis was conducted by a *t*-test. The count data was shown by the number of cases or percentage, and the statistical treatment was performed by a chi-square test. The consistency of the two imaging methods was tested by kappa consistency analysis: kappa≦0.4, poor consistency; 0.4 < kappa≦0.6, general consistency; 0.6 > kappa≦0.8, high consistency; and kappa > 0.8, good consistency.

## 3. Results

### 3.1. Wavelet Entropy Textural Features

Since some entropy values among the 8 wavelet entropy features showed a significantly skewed distribution with widely differing orders of magnitude across features, all features were log-transformed. They were approximately normally distributed and varied within an appropriate range. The log-transformed eigenvectors are denoted as T = [*T*_1_, *T*_2_, *T*_3_, *T*_4_, *T*_5_, *T*_6_, *T*_7_, *T*_8_]. Wavelet entropy results extracted from imaging data of 60 normal subjects and 60 pneumoconiosis patients are shown in Table 1.

### 3.2. Feature Selection

The decision tree constructed with the C 5.0 algorithm is shown in Figure 1. In this decision tree, a total of six features appear at the branches, and thus, the eigenvectors *T* are constructed from these six wavelet entropies.

(8) $$\begin{array}{c} T^{*}=\left[T_{1},T_{2},T_{3},T_{5},T_{6},T_{7}\right]. \end{array}$$

### 3.3. SVM Classification Results

The classification accuracy, sensitivity, and specificity of the SVM classifier models using Gaussian kernel, linear kernel, and polynomial kernel functions, respectively, are shown in Table 2. After feature selection, the classification performance of SVM classifiers with different kernel functions was all improved, indicating that the decision tree algorithm feature selection was helpful to eliminate noisy features and redundant features and improve the performance of classifiers.

From the ROC curves shown in Figure 2, the classification performance of SVM varies when selecting different kernel functions. The classification performance of SVM was related to both the selection of kernel function and the selection of features. Using the selected feature subset, when the linear kernel function of SVM was used, the classification performance was the best. The AUC is 0.90, and the classification accuracy is 84.2%.

The article "Intelligent Image Diagnosis of Pneumoconiosis Based on Wavelet Transform-Derived Texture Features" was published in 2022. Journal: Comput Math Methods Med.

### 3.4. Consistency Analysis

In all 60 cases under High KV DR detection: in 33 cases in stage I, with overall density grade 1 small shadow, distribution range is 2-4 lung areas; in 11 cases in stage II, with overall density grade 2-3 small shadows, distribution range is not less than 4 lung areas; in 8 cases in stage III, large shadow was found. In CT detection, in 40 cases in stage I, grade 1 small density shadow was found; in 12 cases in stage II, grade 2-3 small shadow with or without complications was found; in 8 cases in stage III, large shadow with related complications was found. Typical cases are shown in Figures 3 and 4.

The comparison and analysis of high KV DR and chest CT detection results showed that 51 cases (85.0%) had the same results for pneumoconiosis. Among them, 32 cases (53.0%) were consistent with stage I, 11 cases (18.3%) were consistent with stage II, and 8 cases (13.3%) were consistent with stage III. A kappa consistency test showed that kappa = 0.737 and *P* < 0.001. Details are shown in Figure 5.

### 3.5. Detection Rate of Different Stages

The gold standard was the diagnosis conclusion of the occupational pneumoconiosis expert group. There were 40 stage I cases, the correct detection rate was 80.0% in DR, and there were 7 cases of undetermined diagnosis and 1 case of misdiagnosis as stage III; the correct detection rate was 95.0% in CT, and 2 cases were misdiagnosed as stage III. There was a significant difference in the detection rate of pneumoconiosis between the two methods (*P* = 0.031). There were 12 stage II cases, the correct detection rate was 91.7% in DR, and 1 case was misdiagnosed as stage III; the correct detection rate was 100.0% in CT. There were 8 stage III cases; the correct detection rate in both DR and CT was 100.0%. Details are shown in Figure 6.

## 4. Discussion

Since the 1970s, chest radiograph-based computer-assisted diagnostic studies for pneumoconiosis have been successively carried out at home and abroad, and initial results have been achieved. Yu et al. [18] performed gray level histogram and gray level cooccurrence matrix analysis on DR images to diagnose 300 normal chest radiographs with 125 pneumoconiosis (containing stage III pneumoconiosis) chest radiographs with 87.7%-89.2% accuracy by SVM classifier. Chen et al. [19] evaluated the automated classification of abnormal small shadow on radiographs and calculated its size and density. Compared with the expert identification results, the identification of small shadow results has a false detection rate of 19% and a missed detection rate of 28%. In this study, wavelet entropy texture features were used to diagnose pneumoconiosis which is challenging to diagnose clinically with an accuracy of 84.2% and an AUC of 0.90, demonstrating the value of wavelet entropy texture features in diagnosing early-stage pneumoconiosis using DR chest radiographs.

The article "Intelligent Image Diagnosis of Pneumoconiosis Based on Wavelet Transform-Derived Texture Features" was published in 2022. Journal: Comput Math Methods Med.

When using data mining technology to complete the classification task, the classifier algorithm and the selection of classification features are essential. Due to the complex and diverse classification tasks, there are no universal applicable classification algorithms and parameter setting of the algorithms or even uniform and definite selection criteria. For this reason, many researchers have compared multiple classification algorithms that are more widely used, such as neural networks and SVM. Based on the previous work, we selected SVM as a classifier model to compare the effect of different SVM kernel functions on classification results. The results show that SVM with a linear kernel has the best classification performance. The results illustrate that the choice of the SVM kernel function, as well as the setting of other parameters, is tailored to a specific classification task.

In terms of feature selection, effective feature selection can provide as much information as possible while reducing the number of features, resulting in classification algorithms with faster processing, simpler results, and even superior performance. There are many methods for feature selection, such as the relief method, rough set method, and simulated annealing algorithm. Decision tree algorithms are currently one of the most popular algorithms in data mining techniques with built-in feature selection capabilities. It determines the last enrolled feature by finding the best classification feature that splits the dataset into subsets and loops down until the conditions for the decision tree to stop growing are met. A decision tree is therefore a supervised feature selection method, the results of which are those features that are considered to best satisfy the classification requirements in each subset.

The main pathological changes of occupational pneumoconiosis were silicosis and pulmonary interstitial fibrosis. The main symptoms are chest pain, chest tightness, shortness of breath, and dyspnea. Its early detection and treatment can delay the development of the disease, alleviate the pain of patients, improve the quality of life, and prolong the survival period. Therefore, accurate diagnosis and staging of occupational pneumoconiosis are particularly important [20, 21].

The article "Intelligent Image Diagnosis of Pneumoconiosis Based on Wavelet Transform-Derived Texture Features" was published in 2022. Journal: Comput Math Methods Med.

With the rapid development of medical imaging, chest CT examination technology is gradually widely used in the diagnosis of occupational pneumoconiosis, and its advantages in the diagnosis of pneumoconiosis are gradually highlighted [22, 23]. The high KV DR is an imaging method that uses tube voltage above 120 kV to generate X-ray with high energy in order to obtain rich levels of imaging range. It is usually used for screening and diagnosis of occupational pneumoconiosis. In X-ray photography with voltage above 120 kV, Compton scattering effect dominates the absorption of X-ray in body tissues [24, 25]. The image density of each part of tissue structure is affected by atomic number and body thickness, and the density difference of bone, soft tissue, fat, and gas is reduced correspondingly, so it is commonly used in the general survey and diagnosis of occupational pneumoconiosis. However, the image contrast is reduced and the haze is increased while the rich layers are obtained. In addition, the selection and adjustment of exposure conditions, distance, posture, inspiratory state, artifact, and window technology during high KV DR will also affect the image quality.

The characteristic imaging manifestations of occupational pneumoconiosis are multiple nodular and striped shadows in the lung, enhanced and disordered lung markings, emphysema, thickening of interlobular septum, and some changes in the hilum [26]. However, some reports show that the accuracy of X-ray diagnosis of silicosis is low, and misdiagnosis and missed diagnosis are easy to occur [20]. In this group of data, it was found that 7 cases of stage I pneumoconiosis were not clearly detected in DR. However, the scattered miliary nodules could be observed in the same patient's CT images. The reasons may be as follows: firstly, the density of small nodules in stage I pneumoconiosis is low, and the density is small; secondly, due to the overlapping of ribs, mediastinum, heart, and large vessels and soft tissue, the lung field lesions in the covered part are not well displayed; finally, the image density resolution of DR is low, which can not fully display the shape and density characteristics of the lesions, which is not conducive to observation [27]. The greatest advantage of chest CT is high density resolution, and when CT is used to examine pneumoconiosis, doctors can perform tubular reconstruction and sagittal reconstruction to clearly show the structure of pulmonary lobules and the characteristic changes of pulmonary interstitial fibrosis, including interlobular septal thickening, subpleural line, nodules and honeycomb shadows in interlobular septum, cavities, and calcification in lesions. The lung window and mediastinal window can also be changed for further observation, so the chest CT is more sensitive for the stage I pneumoconiosis. But in the stage II and stage III cases, the diagnosis coincidence rate is very high; there is no significant difference in detection rate between the DR and CT, because the imaging performance of pneumoconiosis patients in this stage has been very obvious, with many lesions and wide range, being easy to observe and analyze, with comprehensive judgment. However, two patients were still diagnosed as stage III by CT and DR at admission, and the diagnosis results were corrected to stage I and stage II, respectively, at discharge. The cause of misdiagnosis was considered that the patients were overstaged because of the imaging interference of pulmonary tuberculosis and pleural thickening. Therefore, it is suggested that in the diagnosis of occupational pneumoconiosis, we should have a higher ability of differential analysis of lung lesions in order to do a good job in differential diagnosis.

The article "Intelligent Image Diagnosis of Pneumoconiosis Based on Wavelet Transform-Derived Texture Features" was published in 2022. Journal: Comput Math Methods Med.

## 5. Conclusions

In summary, it is helpful to improve the early diagnosis level of pneumoconiosis by using SVM to make an intelligent diagnosis based on the wavelet entropy of the image. In addition, the chest CT is better than chest DR in the early diagnosis of occupational pneumoconiosis and complications; the combined application of the two imaging methods can improve the detection rate and accurate staging of occupational pneumoconiosis. Therefore, while the DR is a routine screening and diagnosis of occupational pneumoconiosis, the selective application of chest CT examination can play a good role in diagnosis and supplement.

## Figures and Tables

**Figure 1:** Decision tree used for feature selection.

**Figure 2:** ROC curves of support vector machines for diagnosis of pneumoconiosis.

**Figure 3:** Typical case from a patient with stage I of occupational silicosis. (a) High KV DR show increased and disordered lung markings; small dot shadow is not obvious. (b) CT shows diffuse miliary nodules in both lungs with ground glass-like changes.

**Figure 4:** Typical case from a patient with stage II of occupational silicosis. (a) High KV DR shows scattered small nodules in both lungs, thickened hilum, smooth diaphragm surface, and sharp costophrenic angle. (b) Lung window of CT shows small nodules scattered in all the two lungs, partially fused into a mass; pleural adhesion and thickening were also found. (c) Mediastinal window of CT shows the obvious fusion adhesion between the nodule and pleura.

**Figure 5:** Consistency analysis of high KV DR and CT detection.

The article "Intelligent Image Diagnosis of Pneumoconiosis Based on Wavelet Transform-Derived Texture Features" was published in 2022. Journal: Comput Math Methods Med.

**Figure 6:** Different stages of occupational pneumoconiosis detected by DR and CT.

**Table 1:** Wavelet-based entropy from healthy people and patients with pneumoconiosis.

Wavelet entropy	Healthy	Pneumoconiosis	*P* value
*T*_1_	-0.972	1.154	0.589
*T*_2_	-1.795	3.532	0.176
*T*_3_	-5.192	9.538	<0.001
*T*_4_	-4.036	6.743	0.005
*T*_5_	-2.629	4.341	0.031
*T*_6_	-0.527	0.776	0.754
*T*_7_	-0.254	0.385	0.887
*T*_8_	-1.263	2.246	0.435

**Table 2:** Classification results based on different SVM classifier models (%).

Kernel function	Accuracy (%)		Sensitivity (%)		Specificity (%)	
	Full set	Subset	Full set	Subset	Full set	Subset
Gaussian	78.3	82.5	68.3	73.3	88.3	91.6
Linear	75.8	84.2	61.6	75.0	90.0	93.3
Polynomial	75.8	80.8	60.0	71.6	91.6	90.0

## Data Availability

The data presented in this study are available on request from the corresponding author.

## References

[1] Fan Y., Xu W., Wang Y., Wang Y., Yu S., Ye Q. (2020). Association of occupational dust exposure with combined chronic obstructive pulmonary disease and pneumoconiosis: a cross-sectional study in china. *BMJ Open*.

[2] Han L., Yao W., Bian Z. (2019). Characteristics and trends of pneumoconiosis in the Jiangsu Province, China, 2006^−^2017. *International Journal Environment Research Public Health*.

[3] Zhao J. Q., Li J. G., Zhao C. X. (2019). Prevalence of pneumoconiosis among young adults aged 24-44 years in a heavily industrialized province of China. *Journal of Occupational Health*.

[4] Kurth L., Laney A. S., Blackley D. J., Halldin C. N. (2020). Prevalence of spirometry-defined airflow obstruction in never-smoking working us coal miners by pneumoconiosis status. *Occupational and Environmental Medicine*.

[5] Chiarchiaro J., Tomsic L. R., Strock S. (2018). A case series describing common radiographic and pathologic patterns of hard metal pneumoconiosis. *Respiratory Medicine Case Reports*.

[6] Altınöz H., Çelikkalkan C., Horasan G. D., Hamşioğlu F., Cengiz N., Orbay H. (2016). Socio-demographic and clinical characteristics of turkish workers with pneumoconiosis. *Central European Journal of Public Health*.

[7] Shi P., Xing X., Xi S. (2020). Trends in global, regional and national incidence of pneumoconiosis caused by different aetiologies: an analysis from the global burden of disease study 2017. *Occupational and Environmental Medicine*.

[8] Chen H., Xu N., Zhu F., Ge T., Li Y., Ge J. (2017). Malignant pleural mesothelioma and tuberculous empyema: Ct differential diagnosis. *Journal of Medical Imaging and Health Informatics*.

[9] Wang X., Yu J., Zhu Q. (2020). Potential of deep learning in assessing pneumoconiosis depicted on digital chest radiography. *Occupational and Environmental Medicine*.

The article "Intelligent Image Diagnosis of Pneumoconiosis Based on Wavelet Transform-Derived Texture Features" was published in 2022. Journal: Comput Math Methods Med.

[10] Berk S., Dogan D. O., Gumus C., Akkurt I. (2016). Relationship between radiological (x-ray/hrct), spirometric and clinical findings in dental technicians' pneumoconiosis. *The Clinical Respiratory Journal*.

[11] Zhang L., Wang C., Yan Q., Zhang T., Han Z., Jiang G. (2017). Diagnostic and clinical application value of magnetic resonance imaging (MRI) for progressive massive fibrosis of coal worker pneumoconiosis: case reports. *Medicine (Baltimore)*.

[12] Ding Y., Wei Y., Zhang S., Yu S. (2021). Reversible information of encrypted image based on feature difference detection and wavelet transform. *Contrast Media Mol Imaging*.

[13] Hari L. M., Venugopal G., Ramakrishnan S. (2022). Dynamic contraction and fatigue analysis in biceps brachii muscles using synchrosqueezed wavelet transform and singular value features. *Proceedings of the Institution of Mechanical Engineers. Part H*.

[14] Zhou M., Boyd B. D., Taylor W. D., Kang H. (2021). Double‐wavelet transform for multi-subject resting state functional magnetic resonance imaging data. *Statistics in Medicine*.

[15] Tang Z., Li Y., Chai X., Zhang H., Cao S. (2020). Adaptive nonlinear model predictive control of nox emissions under load constraints in power plant boilers. *Journal of Chemical Engineering of Japan*.

[16] Khoje S. (2018). Appearance and characterization of fruit image textures for quality sorting using wavelet transform and genetic algorithms. *Journal of Texture Studies*.

[17] Chen H., Li W., Zhu Y. (2021). Improved window adaptive gray level co-occurrence matrix for extraction and analysis of texture characteristics of pulmonary nodules. *Computer Methods and Programs in Biomedicine*.

[18] Yu P., Xu H., Zhu Y., Yang C., Sun X., Zhao J. (2011). An automatic computer-aided detection scheme for pneumoconiosis on digital chest radiographs. *Journal of Digital Imaging*.

[19] Chen X., Toriwaki J. -I., Hasegawa J. -I. (1990). Automated classification of pneumoconiosis radiographs based on recognition of small rounded opacities. *Systems and Computers in Japan*.

[20] Okumura E., Kawashita I., Ishida T. (2017). Computerized classification of pneumoconiosis on digital chest radiography artificial neural network with three stages. *Journal of Digital Imaging*.

[21] Ulker O., Yucesoy B., Demir O., Tekin I., Karakaya A. (2008). Serum and bal cytokine and antioxidant enzyme levels at different stages of pneumoconiosis in coal workers. *Human & Experimental Toxicology*.

[22] Choi E. K., Park H. L., Yoo I. R., Kim S. J., Kim Y. K. (2020). The clinical value of f-18 fdg pet/ct in differentiating malignant from benign lesions in pneumoconiosis patients. *European Radiology*.

The article "Intelligent Image Diagnosis of Pneumoconiosis Based on Wavelet Transform-Derived Texture Features" was published in 2022. Journal: Comput Math Methods Med.

[23] Costa C., Ascenti G., Scribano E. (2016). CT patterns of pleuro-pulmonary damage caused by inhalation of pumice as a model of pneumoconiosis from non-fibrous amorphous silicates. *La Radiologia Medica*.

[24] Fauber T. L., Cohen T. F., Dempsey M. C. (2011). High kilovoltage digital exposure techniques and patient dosimetry. *Radiologic Technology*.

[25] Jang J. S., Yang H. J., Koo H. J. (2018). Image quality assessment with dose reduction using high kVp and additional filtration for abdominal digital radiography. *Physica Medica*.

[26] Şener M. U., Şimşek C., Özkara Ş., Evran H., Bursali İ., Gökçek A. (2019). Comparison of the international classification of high-resolution computed tomography for occupational and environmental respiratory diseases with the international labor organization international classification of radiographs of pneumoconiosis. *Industrial Health*.

[27] Guan C. S., Yan S., Lv Z. B. (2020). Ct imaging and pathological basis of linear shadow connecting pulmonary segmental artery to horizontal fissure. *Medicine (Baltimore)*.

